# A circular RNA, circUSP36, accelerates endothelial cell dysfunction in atherosclerosis by adsorbing miR-637 to enhance WNT4 expression

**DOI:** 10.1080/21655979.2021.1964891

**Published:** 2021-09-14

**Authors:** Jian-guo Huang, Xia Tang, Jiang-jie Wang, Jia Liu, Ping Chen, Yan Sun

**Affiliations:** a Department of Vascular Surgery, Linyi Central Hospital, Linyi, Shandong Province, China; b Department of Mental Health, Yishui People’s Hospital, Linyi, Shandong Province, China

**Keywords:** Atherosclerosis, circRNA, miR-637, Wnt4, USP36, endothelial cell

## Abstract

Atherosclerosis is a fatal disorder that is fundamental to various cardiovascular diseases and severely threatens people’s health worldwide. Several studies have demonstrated the role of circular RNAs (circRNAs) in the pathogenesis of atherosclerosis. circUSP36 acts as a key modulator in the progression of atherosclerosis, but the molecular mechanism underlying this role is as yet unclear. This study aimed to elucidate the mechanism by which circUSP36 exerts its function in an in vitro cell model of endothelial cell dysfunction, which is one of pathological features of atherosclerosis. The circRNA traits of circUSP36 were confirmed, and we observed high expression of circUSP36 in endothelial cells exposed to oxidized low-density lipoprotein (ox-LDL). Functional assays revealed that overexpression of circUSP36 suppressed proliferation and migration of ox-LDL-treated endothelial cells. In terms of its mechanism, circUSP36 adsorbed miR-637 by acting as an miRNA sponge. Moreover, enhanced expression of miR-637 abated the impact of circUSP36 on ox-LDL-treated endothelial cell dysregulation. Subsequently, the targeting relationship between miR-637 and WNT4 was predicted using bioinformatics tools and was confirmed via luciferase reporter and RNA pull-down assays. Notably, depletion of WNT4 rescued circUSP36-mediated inhibition of endothelial cell proliferation and migration. In conclusion, circUSP36 regulated WNT4 to aggravate endothelial cell injury caused by ox-LDL by competitively binding to miR-637; this finding indicates circUSP36 to be a promising biomarker for the diagnosis and therapy of atherosclerosis.

## Introduction

Atherosclerosis, a chronic inflammatory disorder, is fundamental for the vast majority of cardiovascular diseases, including coronary heart disease, myocardial infarction, and ischemic stroke, and it clinically manifests as arterial lipid deposition and fibrinogen accumulation [1,2]. Atherosclerosis remains one of the most lethal diseases worldwide, causing over 20 million deaths and accounting for approximately 84.5% of cases of cardiovascular disease; thus, atherosclerosis a distressing global public health concern [3–5]. The pathogenesis of atherosclerosis is extremely complicated and involves diverse factors, such as genes, obesity, hyperlipidemia, smoking, and environmental factors [6,7]. Hence, a comprehensive elucidation of its pathogenesis would be helpful for identifying potent diagnostic indicators and therapeutic strategies.

Endothelial cells are the basic components of the cardiovascular system and play a crucial role in maintaining vascular homeostasis [8]. Endothelial cell dysfunction is one of the most common pathological features of atherosclerosis onset and development [9]. Oxidized low-density lipoprotein (ox-LDL) has been identified as an important contributor to the pathogenesis of atherosclerosis; it induces endothelial damage characterized by aberrant cell proliferation, cell migration, apoptosis, inflammation, and angiogenesis, thereby destroying endothelial integrity and exacerbating lipid deposition [10,11]. An increasing number of studies have demonstrated the use of endothelial cells subjected to ox-LDL treatment as a cell model for atherosclerosis [12–14]. Accordingly, the identification of key regulators in the dysfunction of endothelial cells is urgently needed to improve the treatment of atherosclerosis.

Circular RNAs (circRNAs), which have drawn the attention of researchers in recent years, comprise a type of non-coding RNA and possess a covalently closed-loop structure without a free 5′ cap or 3′ tail via back-splicing [15,16]. In addition, circRNAs exhibit ubiquitous expression in eukaryotic cells and are more stable than their linear mRNAs [17]. These traits suggest the possibility of using circRNAs as potential indicators in the diagnosis and treatment of human diseases [18]. Numerous studies have revealed that circRNAs participate in the initiation and progression of atherosclerosis through the regulation of cell function. For instance, circHIPK3 functions as a modulator of atherosclerosis development by affecting endothelial cell behavior and autophagy [19]. circCHFR contributes to vascular smooth muscle cell proliferation and migration in atherosclerosis by targeting the miR-370/FOXO1/Cyclin D1 axis [20]. CircRSF1 facilitates cell proliferation, migration, and tube formation in ox-LDL-treated endothelial cells via the miR-758/CCND2 pathway in atherosclerosis [21]. Thus, it is increasingly important to explore the role of circRNAs in atherosclerosis. circUSP36 (also known as circ_0003204) has been reported to be prominently upregulated among the top 10 differentially expressed circRNAs in human umbilical vein endothelial cells administered ox-LDL [22], but the mechanism of its function has not yet been exhaustively elucidated.

In our study, we hypothesized that circUSP36 promotes atherosclerosis by inducing the proliferation and migration of ox-LDL-treated endothelial cells. The aim of the current study was to verify the expression pattern and functional role of circUSP36 in ox-LDL-treated endothelial cells. More importantly, we intended to provide novel insights into the potential mechanism underlying the role of circUSP36 in ox-LDL-induced endothelial cell dysfunction.

## Materials and methods

### Cell culture and treatment

Human aortic endothelial cells acquired from ATCC (Manassas, VA, USA) were maintained in DMEM (Gibco, Carlsbad, CA, USA) supplemented with 10% fetal bovine serum (FBS; Hyclone, Logan, UT, USA), 1% endothelial cell growth factor (ScienCell, Carlsbad, CA, USA), and 1% penicillin-streptomycin (Hyclone). Endothelial cells were cultivated at 37°C in an atmosphere of 5% CO_2_. To simulate endothelial cell dysfunction in vitro, endothelial cells were exposed to 100 µg/ml ox-LDL (Sigma, St. Louis, MO, USA) for 24 h, as described previously [23].

### RNase R and actinomycin D treatment

The stability of circUSP36 was detected by the RNase R and actinomycin D assays [24]. To conduct RNase R treatment, 2 mg total RNA from endothelial cells was incubated for 0.5 h with or without 5 U/mg RNase R. For the actinomycin D assay, endothelial cells were treated with 2 μg/ml actinomycin D for different time periods (0, 4, 8, and 12 h). Next, the expression of circUSP36 and linear RNA was analyzed by polymerase chain reaction (PCR).

### Cell transfection

circUSP36-overexpression vectors were constructed by cloning the transcript sequence of circUSP36 into pcDNA3.1 plasmids obtained from Genepharma (Shanghai, China). Small interfering RNAs (siRNA) against WNT4 or circUSP36 for knockdown of WNT4 or circUSP36 (named as si-WNT4 and si-circUSP36, respectively) and their negative control the scramble siRNA (named as si-NC) were designed and supplied by RiboBio Co., Ltd. (Guangzhou, China). To regulate miR-637 expression, oligonucleotides including miR-637 mimic and inhibitor, as well as their corresponding mimic NC and inhibitor NC, were acquired from Genepharma. Cell transfection was performed using Lipofectamine 2000 (Invitrogen, Carlsbad, CA, USA) according to the instructions [25].

### Quantitative real-time PCR (qRT-PCR)

Total RNA derived from endothelial cells was isolated using TRIzol reagent (Invitrogen) [24]. Reverse transcription was performed using Superscript II reverse transcriptase (Invitrogen), according to the manufacturer’s instructions. Afterward, qRT-PCR was conducted with SYBR Green Real-time PCR Master Mix (Takara, Dalian, China) on an ABI Prism 7500 Real-time PCR System (Applied Biosystems, Foster City, CA, USA). The expression of circUSP36 and WNT4 was normalized to that of GAPDH, and miR-637 expression was normalized to that of U6. All experimental data were analyzed using the 2^−ΔΔCt^ method.

### Cell proliferation assay

A cell counting kit 8 (CCK-8) assay was performed to determine endothelial cell proliferation [26]. Following the manufacturer’s guidelines, 5 × 10^3^ endothelial cells were plated in each well of a 96-well plate and cultured for 12, 24, 48, and 72 h at 37°C. Then, endothelial cells were treated with 10 μl CCK-8 (Dojindo, Shanghai, China) and incubated for another 2 h. The optical density was measured at a wavelength of 450 nm with a microplate reader (Bio-Rad Laboratories, Inc., Hercules, CA, USA).

### Transwell assay

Transwell assays were performed to measure cell migration using Transwell chambers (Corning, Cambridge, MA, USA) [27]. Following the corresponding processing, 2 × 10^4^ endothelial cells were harvested, resuspended in DMEM without serum, and placed into the apical chamber. The lower chamber was filled with DMEM containing 10% FBS. 20 h later, the endothelial cells that passed through the filter were fixed with 4% methanol, stained with 1% crystal violet (Beyotime, Beijing, China) and counted in five random fields using a microscope (100×; Olympus, Tokyo, Japan).

### Wound healing assay

Cell migration ability was evaluated using a wound healing assay [26]. In short, endothelial cells were cultured until 90% confluence, and subsequently, a scratch was made using a sterile 100-μl pipette tip. Cells were monitored and photographed under a microscope at 0 and 48 h after the cells were wounded. The scratch distance was measured using Image-Pro Plus software.

### RNA pull-down

Biotinylated miR-637 and miR-NC were obtained using the Pierce RNA 3ʹ End Desthiobiotinylation Kit (Thermo Fisher Scientific, Boston, MA, USA) according to the instructions [25]. Endothelial cells were transfected with biotin-labeled miRNAs for 48 h; the collected cells were lysed using cell lysis buffer (Invitrogen), incubated with streptavidin magnetic beads, and subjected to qRT-PCR analysis.

### *Fluorescence* in situ *hybridization (FISH)*

The FISH assay was carried out with a Fluorescent *in situ* Hybridization Kit (RiboBio Co., Ltd.) in accordance with the instructions [28]. Briefly, after fixation, endothelial cells were treated with 0.5% Triton X-100, dehydrated, and hybridized with Alexa 488-labeled circUSP36 probes and Cy3-labeled miR-637 probes. Thereafter, endothelial cells were rinsed with 2× SSC buffer and counterstained with DAPI (Sigma). Images were captured using a confocal microscope (Leica, Wetzlar, Germany).

### Luciferase reporter gene assay

The wild-type and mutant sequences of circUSP36 were ligated into the luciferase reporter plasmid psiCHECK-2 (Promega, Madison, WI, USA) to synthesize circUSP36-WT and circUSP36-MUT [27]. WNT4-WT and WNT4-MUT constructs were acquired using the same method. HEK-293 T cells were co-transfected with miR-637 mimic or negative control mimic NC, and luciferase reporter plasmids were constructed using Lipofectamine 2000. After 24 h, a dual-luciferase reporter system (Promega) was used to detect luciferase activity according to the manufacturer’s instructions.

### Western blotting

Protein isolation was carried out using RIPA buffer (Thermo Fisher Scientific), and a bicinchoninic acid assay kit (Thermo Fisher Scientific) was used for protein quantitation [27]. Protein samples were separated by 10% SDS-PAGE and transferred to polyvinylidene fluoride membranes (Millipore, Billerica, MA, USA). After blocking in 5% defatted milk, PVDF membranes were probed with primary antibodies for WNT4 or GAPDH at 4°C overnight, incubated with HRP-conjugated secondary antibody at room temperature for 4 h, and visualized using an ECL kit on the ChemiDoc™ MP Imaging System (Bio-Rad Laboratories, Inc.)

## Statistical analysis

All results are shown as mean ± standard deviation (SD), and data processing was conducted using SPSS (version 19.0; IBM Corp., Armonk, USA). Differences between two groups were analyzed using unpaired Student’s *t*-tests. Comparison of data among three or more groups was performed using ANOVA. Statistical significance was set at *p* < 0.05.

## Results

In this study, we use endothelial cell dysfunction as an in vitro cell model for studying atherosclerosis, and intend to clarify the important role of circUSP36. Studies have found that circUSP36 may be a promising biomarker for the diagnosis and treatment of atherosclerosis. We hypothesize that circUSP36 can promote the development of atherosclerosis by promoting endothelial cell dysfunction. Overexpression of circUSP36 inhibited the proliferation and migration of endothelial cells treated with oxLDL. The enhanced expression of miR-637 alleviated the effect of circUSP36 on the dysregulation of endothelial cells treated with ox-LDL. circUSP36 regulates WNT4 by competitively binding miR-637, aggravating atherosclerotic endothelial cell damage caused by ox-LDL.

### circUSP36 expression was upregulated in ox-LDL-treated endothelial cells

To identify the characteristics of circUSP36 in endothelial cells, circUSP36 was first subjected to RNase R treatment. circUSP36 exhibited a greater resistance to RNase R digestion compared to its linear mRNA (Figure 1a). Next, qRT-PCR analysis showed that the stability of circUSP36 was much higher than that of the USP36 linear isoform in endothelial cells treated with actinomycin D, further confirming the loop structure of circUSP36 (Figure 1b). Corroborating the above results, the existence of circUSP36 was only detected by qRT-PCR using cDNA rather than gDNA as the template (Figure 1c). Considering that ox-LDL treatment is widely used to simulate pathological features of atherosclerosis in vitro [29], ox-LDL-treated endothelial cells were used to verify the expression profile of circUSP36. The results of qRT-PCR revealed that the expression of circUSP36 was overtly elevated in endothelial cells exposed to ox-LDL (Figure 1d). These findings validated the circular features of circUSP36 and high circUSP36 expression levels in ox-LDL-treated endothelial cells.

**Figure 1.** **circUSP36 expression was upregulated in ox-LDL-treated endothelial cells**. (a) qRT-PCR analysis for circUSP36 expression in endothelial cells treated with or without RNase R digestion (n = 3). (b) qRT-PCR detection of circUSP36 and linear mRNA in endothelial cells exposed to Actinomycin D (n = 3). (c) Divergent primers could amplify circUSP36 in cDNA but not gDNA (n = 3). (d) circUSP36 expression in endothelial cells treated with or without ox-LDL was detected via use of qRT-PCR assay (n = 3). **P < 0.01

### Ectopic expression of circUSP36 attenuated endothelial cell proliferation and migration

We attempted to illustrate the function of circUSP36 in endothelial cells treated with ox-LDL. circUSP36 was overexpressed to conduct gain-of-function assays and qRT-PCR analysis confirmed that cells transfected with circUSP36-overexpression vectors presented high expression of circUSP36 (Figure 2a). The CCK-8 assay revealed that enforced expression of circUSP36 caused a remarkable decrease in endothelial cell viability (Figure 2b). Additionally, the transwell assay demonstrated that the number of migrated endothelial cells was reduced when circUSP36 was upregulated (Figure 2c-d). Consistently, the wound healing assay indicated that the migration capacity of endothelial cells was restrained by overexpression of circUSP36 (Figure 2e). These results prove that circUSP36 attenuates endothelial cell dysfunction and may alleviates the development of atherosclerosis in vitro.

**Figure 2.** **Ectopic expression of circUSP36 attenuated endothelial cell proliferation and migration**. (a) The efficiency of circUSP36 overexpression was examined by qRT-PCR (n = 3). (b) CKK-8 assay explored the viability of ox-LDL-treated endothelial cells in different groups (n = 6). (c-e) Transwell and wound-healing assays measured the migration ability of endothelial cells exposed to ox-LDL for the indicated times after transfection (n = 6). Cells migrating to the underside of the transwell insert were counted. **P < 0.01

### circUSP36 adsorbed miR-637 in a sponge form

Given that circRNAs can act as sponges for miRNAs in atherosclerosis [30], we aimed to clarify the pathway by which circUSP36 executes its function. Therefore, using the circInteractome database, miR-637 was found to be a predicted miRNA target of circUSP36. As shown in Figure 3a, circUSP36 harbored potential miR-637 binding sites. The luciferase activity of HEK-293 T cells was impaired only by co-transfection of miR-637 mimic and wild-type circUSP36 (Figure 3b). qRT-PCR analysis suggested that knockdown of circUSP36 enhanced the expression of miR-637, whereas overexpression of circUSP36 led to a decrease in miR-637 levels (Figure 3c). In addition, the RNA pull-down assay revealed that the expression of circUSP36 was abundant in the miR-637 pull-down complex, which further confirmed that circUSP36 binds to miR-637 (Figure 3d). Subsequently, the localization of circUSP36 and miR-637 in endothelial cells was determined using FISH. circUSP36 and miR-637 were preferentially expressed in the cytoplasm of endothelial cells (Figure 3e). Overall, these results indicate that circUSP36 is an miRNA sponge for miR-637.

**Figure 3.** **circUSP36 adsorbed miR-637 in a sponge form**. (a) Binding sites between circUSP36 and miR-637 as predicted by circInteractome. (b) Interaction between circUSP36 and miR-637 was evaluated with a luciferase reporter assay (n = 3). (c) Effects of circUSP36 on miR-637 expression were assessed by qRT-PCR (n = 3). (d) RNA pull-down assay tested the binding affinity between circUSP36 and miR-637 (n = 3). (e) FISH was conducted for the co-localization of circUSP36 and miR-637 in endothelial cells (n = 3). **P < 0.01

### Overexpression of miR-637 relieved the role of circUSP36 in endothelial cells

To elucidate the potential of miR-637 in atherosclerosis progression, miR-637 expression was repressed in ox-LDL-treated endothelial cells following transfection with circUSP36-overexpression vectors. qRT-PCR analysis confirmed the transfection efficiency of the miR-637 mimic (Figure 4a). Cell proliferation in circUSP36-overexpressing endothelial cells was recovered by the enhanced expression of miR-637 (Figure 4b). Moreover, the miR-637 mimic restored cell migration ability, which was weakened by upregulation of circUSP36 (Figure 4c-d). Similarly, the wound healing assay verified the role of miR-637 in circUSP36-mediated endothelial cell migration (Figure 4e-f). The above findings provide strong evidence that circUSP36 plays a regulatory role in endothelial cell behavior by adsorbing miR-637.

**Figure 4.** **Overexpression of miR-637 relieved the role of circUSP36 in endothelial cells**. (a) Overexpression efficacy of miR-637 mimic was assessed by qRT-PCR (n = 3). (b) Cell proliferation in four different groups was examined with the CCK-8 assay (n = 6). (c-f) Cell migration in four different groups was estimated by transwell and wound-healing assays (n = 6). Cells migrating to the underside of the transwell insert were counted. **P < 0.01

### WNT4 functioned as a downstream target of miR-637

By browsing the targetscan website, WNT4 was found to have a potential affinity for miR-637 (Figure 5a). WNT4 was chosen for subsequent experiments because it has been reported to be involved in the proliferation and migration of endothelial cells [31]. To justify the bioinformatics prediction, a luciferase reporter gene assay was performed. We noticed that the miR-637 mimic lowered the luciferase activity of HEK-293 T cells transfected with the luciferase reporter vector psiCHECK-2 containing the wild-type WNT4 3′ untranslated region (UTR) but had no effect on that of the mutant group (Figure 5b). qRT-PCR analysis and western blotting showed that overexpression of miR-637 dramatically mitigated the mRNA and protein expression levels of WNT4, while miR-637 suppression triggered the opposite outcomes (Figure 5c). In agreement with these findings, WNT4 was significantly enriched by biotin-labeled miR-637 than by biotin-labeled miR-NC (Figure 5d). Thus, these results together confirm the relationship between miR-637 and WNT4.

**Figure 5.** **WNT4 functioned as a downstream target of miR-637**. (a) Binding sequences of miR-637 in WNT4 3ʹ UTR. (b) Luciferase reporter assay was employed to validate the targeting relationship between miR-637 and WNT4 (n = 3). (c) qRT-PCR and western blotting detection of WNT4 expression in endothelial cells transfected with miR-637 mimic/inhibitor or their negative controls (n = 3). (d) Interplay between miR-637 and WNT4 was estimated by the RNA pull-down assay (n = 3). **P < 0.01

### WNT4 was responsible for the effects of circUSP36 on endothelial cell behavior

Lastly, we investigated whether circUSP36 acts as a regulator of atherosclerosis by targeting miR-637-mediated WNT4. We observed that the level of WNT4 was decreased by circUSP36 overexpression and was regained on silencing of WNT4 in ox-LDL-treated endothelial cells (Figure 6a). As expected, the results of the CCK-8 assay showed that knocking out WNT4 can increase the decreased cell viability caused by overexpression of circUSP36 (Figure 6b). The transwell assay indicated that the inhibition of endothelial cells resulting from enhanced expression of circUSP36 was abolished when WNT4 was silenced (Figure 6c-d). Likewise, the wound healing assay demonstrated that downregulation of WNT4 abrogated the impact of circUSP36 on the migration capability of endothelial cells (Figure 6e-f). Thus, we concluded that WNT4 mediates the role of circUSP36 in an *in vitro* cell model of atherosclerosis.

**Figure 6.** **WNT4 was responsible for effects of circUSP36 on endothelial cell behavior**. (a) qRT-PCR detection of WNT4 expression in endothelial cells following different treatments (n = 3). (b) CCK-8 analysis for testing cell proliferation in different groups (n = 6). (c-f) Ability of ox-LDL-treated endothelial cells to migrate was assessed by transwell and wound-healing experiments. (n = 6) Cells migrating to the underside of the transwell insert were counted. **P < 0.01

## Discussion

Atherosclerosis is a leading cause of human mortality globally because of its growing rates of morbidity and fatality [32,33]. Recently, the prevention and treatment of atherosclerosis has attracted increasing attention in the field of medical research [34]. The multifactorial pathophysiological process of atherosclerosis is complex and involves endothelial cell injury, vascular smooth muscle cell differentiation, lipid infiltration, fibrosis, and inflammatory cytokine secretion [12,35–37]. This study focused on the mechanisms underlying endothelial dysfunction. Since ox-LDL is a vital inducer of atherosclerosis progression [38], we used endothelial cells exposed to ox-LDL for *in vitro* studies.

Numerous studies provide strong evidence that circRNAs play a critical role in the occurrence and development of atherosclerosis [39–41]. Abnormal circRNA expression has been shown to be closely associated with atherosclerosis progression [42,43]. A previous report confirmed that circUSP36 was markedly upregulated in ox-LDL-treated endothelial cells through circRNA microarray analysis [22]. Furthermore, the potential of circUSP36 has been explored in the regulation of endothelial cell dysfunction. It has been proven that circUSP36 aggravates endothelial injury caused by ox-LDL by restraining cell proliferation, migration, invasion, and angiogenesis, while promoting apoptosis and inflammation [44–47]. In concert with these previous findings, this study demonstrated that circUSP36 was highly expressed in ox-LDL-treated endothelial cells than in the control group and that enforced expression of circUSP36 suppressed cell proliferation and migration in ox-LDL-treated endothelial cells. These results confirmed that circUSP36 plays a role in the pathogenesis of atherosclerosis.

Overwhelming evidence indicates that the competing endogenous RNA (ceRNA) mechanism is a classical pathway by which circRNAs function in the physiological and pathological processes of atherosclerosis [48,49]. Increasing evidence suggests that circRNAs can act as ceRNAs to protect target genes from miRNA degradation by sponging miRNA [50,51]. Thus, we speculated that circUSP36 is likely to affect endothelial cell dysfunction via the ceRNA mechanism. Through application of the circInteractome database, miR-637 was predicted to be a target of circUSP36. In view of the inhibitory role of miR-637 in atherosclerosis [52], we selected miR-637 as a research object in subsequent explorations of the molecular mechanism. Luciferase reporter gene and RNA pull-down assays validated that miR-637 directly binds to circUSP36. Notably, FISH analysis showed the co-localization of circUSP36 and miR-637 in the cytoplasm of endothelial cells, indicating the potential of circUSP36 as a ceRNA. Moreover, experimental data revealed that overexpression of miR-637 alleviated endothelial damage exacerbated by circUSP36 in ox-LDL-treated endothelial cells. Next, we identified WNT4 as the downstream effector of miR-637 by using bioinformatics analysis. The upregulation of WNT4 has been reported to be strongly related to vascular stenosis, and WNT4 might represent a therapeutic target for the prevention of vascular restenosis in atherosclerosis [53,54]. Consequently, we investigated the interplay between miR-637 and WNT4. As expected, WNT4 served as a target gene for miR-637. Additionally, knockdown of WNT4 offset the role of circUSP36 in ox-LDL-treated endothelial dysfunction in atherosclerosis.

## Data Availability

All the data is available from the corresponding author due to reasonable request

## Highlights

circUSP36 expression was upregulated by ox-LDL-treated

Overexpression of circUSP36 promoted endothelial cell dysfunction

Overexpression of miR-637 relieved the function of circUSP36

WNT4 as a downstream target of miR-637
